RETRACTED

# Diagnostic Effectiveness of Dual Source Dual Energy Computed Tomography for Benign and Malignant Thyroid Nodules

**DOI:** 10.1155/2022/2257304

**Published:** 2022-08-17

**Authors:** Tong Zhu, Kanglin Xie, Chongxiao Wang, Linkui Wang, Wei Liu, Faping Zhang

**Affiliations:** Anhui Wannan Rehabiltation Hospital The Fifth People's Hospital of Wuhu, Radiology Department, Wuhu, China

## Abstract

**Objective:**

To evaluate the diagnostic effectiveness of dual source dual energy computed tomography (DS-DECT) for benign and malignant thyroid nodules.

**Methods:**

Between January 2019 and December 2021, 60 patients with surgically and pathologically verified thyroid nodules treated at our institution were recruited. DS-DECT was administered to all patients. The iodine content of lesioned and normal tissues, the normalized iodine concentration (NIC) and standardized CT values of benign and malignant nodules, the consistency of examination results and pathological findings, and diagnostic effectiveness were all investigated.

**Results:**

The diagnosis accuracy was the same as that of surgical pathology, producing a 100% accuracy for the 60 patients with thyroid nodules (42 were benign and 18 were malignant). The iodine content of lesioned solid tissue differed significantly from that of normal tissue, as did the iodine content of malignant and benign nodules (*P* < 0.05). In the arterial phase, no significant difference was found in NIC and standardized CT values between benign and malignant nodules (*P* > 0.05). The optimal critical NIC for differentiating benign and malignant nodules in the venous phase was 0.74 and the standardized CT value was 0.79 HU according to the receiver operating characteristics (ROC) curve. Malignant nodules were diagnosed when the NIC was <0.74 and the standardized CT value was <0.79 HU, with AUC values of 0.89 and 0.93, respectively, where the sensitivity and specificity of the differential diagnosis of NIC were 90.48% (38/42) and 88.89% (16/18), respectively, and those of the differential diagnosis of standardized CT value were 92.86% (39/ 42) and 94.44% (17/18), respectively. The diagnosis accuracy of DS-DECT was 100%, and the diagnostic results of morphological characteristics and pathological testing were consistent. The sensitivity and specificity of the NIC values and standardized CT values in the venous phase differential diagnosis of benign and malignant nodules were compatible with the morphological differential diagnosis.

**Conclusion:**

DS-DECT is highly accurate in determining the benignity and malignancy of thyroid nodules and has a strong potential for clinical promotion to allow for prompt treatment.

## 1. Introduction

Thyroid nodules are abnormal masses of tissue structure in the thyroid gland and differ significantly from normal thyroid tissue [1]. Thyroid nodules have been more common in China in recent years, and the major causes of thyroid nodules include inflammation and a bad lifestyle. The treatment for thyroid nodules of various types varies greatly [2, 3], with medical treatment as the mainstay for benign nodules and surgical management for malignant ones. For thyroid nodules, regular follow-up, surgery, radioelectric therapy, laser/radiofrequency/microwave ablation, and thyroid hormone suppression are all available clinically, yet no standard treatment protocol has been established [4]. Thyroid nodules belong to the category of “gall disease” in traditional Chinese medicine (TCM) and are often treated clinically with evidence-based treatment to soften and disperse the nodules [5].

RETRACTED

The current diagnostic modalities comprise mainly imaging, immunoassays, and biopsies [6, 7]. Fine-needle aspiration cytology biopsy is the main method for qualitative diagnosis of thyroid nodules, but it is invasive and results in poor patient compliance. Thus, further exploration of safer and more effective diagnostic options is required. Ultrasound and contrast-enhanced CT currently deliver rapid and accurate examinations in the imaging diagnosis of thyroid nodules [8]. Dual-source CT features the advantage of dual-energy imaging with a unique algorithm that separates iodine from soft tissue [9].

Computed tomography energy spectral imaging can acquire various quantitative parameters on the basis of conventional imaging, analyze lesions with the aid of three-dimensional regions of interest, and effectively clarify the internal spatial heterogeneity of lesions, so it has been widely used in the diagnosis of tumor diseases [10]. In addition, dual-source CT compares the iodine content of thyroid nodules and surrounding normal thyroid tissue, displays the CT values of different tissues and organs and lesions, and constructs energy spectrum curves to achieve the judgment of benign and malignant nodules [11, 12]. In addition, it can effectively reflect the state of distribution of base materials such as water, iodine, and calcium and further reflect the margins and internal structure of the lesion with the help of standardized iodine concentration [13]. Herein, this study was conducted to evaluate the diagnostic effectiveness of dual-source dual energy computed tomography (DS-DECT) for benign and malignant thyroid nodules.

## 2. Materials and Methods

### 2.1. Participants

A total of 60 patients with surgically and pathologically confirmed thyroid nodules treated in our hospital between January 2019 and December 2021 were recruited, including 35 males and 25 females, aged 29–78 (52.64 ± 14.42) years. After surgery and a puncture biopsy, the patients were found with thyroid nodules, 42 of which were benign and 18 of which were malignant. The eligible patients and their families were notified about the trial, and they agreed to participate. Patients with functional impairment of vital organs and inability to communicate were excluded. Informed consent was obtained from patients and signed prior to enrollment in this study. The study protocol was approved by the hospital ethics committee. Ethics number: HX-YEYI20190104. All processes were in accordance with the Declaration of Helsinki ethical guidelines for clinical research.

RETRACTED

### 2.2. Methods

The CT scans were performed using the 2nd generation Siemens Dual Source CT (Definition Flash) instrument. Before the examination, the patient was informed about the relevant examination precautions. The patient was injected with 70–90 ml of non-ionic contrast agent iohexol (300 mg/ml) at a rate of 3 ml per second with the CT machine in the dual energy mode and tube voltages of 80 and 140 kV. Body thickness and density were adjusted before the examination with a layer thickness of 5 mm. A CT plain scan was performed, the patient's axial raw data were analyzed, and then the data were reconstructed with a reconstructed layer thickness of 0.75 mm. The 3D software was applied to obtain image information in the coronal and sagittal planes, and the scan was performed from the skull base to the thoracic inlet. The patient was kept in a supine position during the scan to avoid the influence of clavicular artifacts on the examination results. After routine scanning, a contrast-enhanced scan was performed at 30 and 60 seconds after the contrast injection in the dual-energy mode to obtain the DS-DECT images.

#### 2.2.1. Measurement of Iodine Content

The iodine content of the region of interest (ROI) was measured by a double-blind method in the iodine images, with the solid part of the ROI selected, avoiding calcifications and artifacts, in the range of 10 mm 2 to 20 mm 2, and the averaged value was obtained from three measurements.

#### 2.2.2. Diagnostic Criteria

Lesions with regular morphology, clear borders, and no “intensification residual circle sign” in the contrast scan are considered benign nodules. Lesions with irregular morphology, blurred boundary, microcalcifications inside, “reinforced residual circle sign” in the contrast scan and enlarged lymph nodes in the neck were considered malignant nodules.

During the examination, the CT signs were analyzed to determine the nature of the nodule. Malignant nodules show disruption of the pseudo-envelope to form an interrupted reinforcing ring, which completely penetrates the envelope and invades the surrounding tissue.

RETRACTED

### 2.3. Observation Indices

1. Iodine content of diseased solid and normal tissues was compared.
2. Normalized iodine concentration (NIC) and standardized CT values of benign and malignant nodules: NIC and standardized CT values were calculated for benign and malignant nodules. NIC = intra-lesion iodine concentration/intra-phase carotid iodine concentration; standardized CT value = intra-lesion CT value/intra-phase carotid CT value.
3. Consistency between examination results and pathological results: Consistency analysis was performed using the Kappa test, with Kappa < 0.2 for poor consistency, 0.2 ≤ Kappa < 0.4 for fair consistency, 0.4 ≤ Kappa < 0.6 for moderate consistency, 0.6 ≤Kappa < 0.8 for good consistency, and 0.8 ≤Kappa ≤ 1 for excellent consistency.
4. Diagnostic efficacy.

### 2.4. Statistical Analysis

SPSS20.0 was adopted for data analyses. The Shapiro–Wilk line normal distribution test was used for the measurement data. Normally distributed measures were expressed as (mean plus or minus standard deviation). Comparisons of means between the two groups were first performed with the chi-squared *F*-test, and data with chi-squared were subjected to the independent samples *t*-test, and data with non-chi-squared were tested with the independent samples *t*-test. Within-group pre-post comparisons were performed with paired-sample *t*-tests. Differences with *P* < 0.05 was considered statistically significant.

## 3. Results

### 3.1. Analysis of Iodine Content in Diseased Solid Tissues and Normal Tissues

Iodine concentration was substantially reduced in sick thyroid tissues compared to normal tissues, as well as significantly lower in malignant nodules compared to benign nodules (*P* < 0.05) (Table 1).

### 3.2. NIC and Standardized CT Values for Benign and Malignant Nodules

There was no significant difference in the arterial phase between NIC and standardized CT readings of benign and malignant nodules (*P* > 0.05). The NIC and normalized CT values of benign nodules were greater in the venous phase than those of malignant nodules (*P* < 0.05) (Table 2).

### 3.3. Examination Results and Pathological Findings

Of the 60 patients with thyroid nodules, 42 cases were benign and 18 cases were malignant.

#### 3.3.1. Morphology

8 out of 42 patients with benign lesions had irregular morphology, and 10 out of 18 patients with malignant nodules had irregular morphology. The detection rate of malignant nodules with irregular morphology (55.56%) was higher than that of benign nodules (19.05%) (*P* < 0.05). The examination results were consistent with the pathological findings, and the diagnostic accuracy of DS-DECT was 100%.

RETRACTED

#### 3.3.2. Boundaries

Distinct lesion margins were found in 42 individuals with benign nodules, with one having a nodule extending into the mediastinum and a clear fat gap between the lesion tissue and surrounding tissues. The boundaries between the lesion tissue and the surrounding tissue were blurred in eighteen cases with malignant lesions. Benign nodular lesions with clean borders were detected at a considerably greater rate than malignant nodules (*P* < 0.001).

#### 3.3.3. Calcification

30 of the 42 individuals with benign lesions had calcification of the lesions, with spotty, eggshell, and massive calcifications being the most common. Five of the 18 patients with malignant tumors had calcification, most of which was fine granular calcification. The detection rate of calcification in benign nodules (71.43%) was significantly higher than that of calcification in malignant nodules (27.78%) (*P* < 0.05) (Table 3 and Figures 1 and 2).

### 3.4. Diagnostic Efficacy

The optimal critical NIC for differentiating benign and malignant nodules in the venous phase was 0.74 and the standardized CT value was 0.79 HU according to the receiver operating characteristics (ROC) curve. Malignant nodules were diagnosed when the NIC was <0.74 and the standardized CT value was <0.79 HU, with AUC values of 0.89 and 0.93, respectively, where the sensitivity and specificity of the differential diagnosis of NIC were 90.48% (38/42) and 88.89% (16/18), respectively, and those of the differential diagnosis of standardized CT value were 92.86% (39/42) and 94.44% (17/18), respectively. The diagnostic results of morphological features and pathological examination were consistent, and the diagnostic accuracy of DS-DECT was 100%. The sensitivity and specificity of the NIC values and standardized CT values in the differential diagnosis of benign and malignant nodules in the venous phase were consistent with the sensitivity and specificity of the morphological differential diagnosis (Kappa = 0.901, 0.883) (Figure 3).

## 4. Discussion

In recent years, the incidence of thyroid nodules has increased significantly with the increased work pressure and changes in the lifestyle of people. Its pathogenesis is mainly associated with abnormal iodine intake, immunity, lipid metabolism, genetics, and other factors, with the core mechanism being the negative feedback regulation of the hypothalamic-pituitary-thyroid axis by many factors leading to the hyperplasia of thyroid follicles and the formation of thyroid nodules [14, 15]. Thyroid nodules generally show no specific clinical manifestations, and patients with abnormal functional manifestations are mostly treated with levothyroxine sodium tablets [16]. However, Western medication predisposes patients to adverse events such as metabolic organ damage and increased pain.

RETRACTED

In TCM, the occurrence of thyroid nodules is considered to be closely related to emotional abnormalities, diet, and loss of proper water and soil [17]. The increased work pressure and accelerated pace of life lead to the loss of spleen health and function and result in the development of nodules, so the treatment should be based on draining the liver and Qi, strengthening the spleen, resolving phlegm, activating blood circulation, and eliminating galls [18, 19]. The nature of benign and malignant thyroid nodules is usually determined by morphology, number, and blood supply on plain or contrast CT scans [20]. In contrast to benign thyroid nodules, malignant thyroid nodules usually appear hypodense because the tumor cells destroy the iodine storage units of the normal thyroid gland. Because of the infiltrative growth of the lesions, the nodules are irregular in shape and the tumor tissue often invades the fibrous envelope. Some malignant tumors may undergo cystic necrosis, such as papillary thyroid carcinoma characterized by cystic changes and calcified wall nodules [21]. Although CT of benign and malignant thyroid nodules shows certain morphological and enhancing features, there are overlaps in conventional imaging presentations, resulting in difficult qualitative diagnosis. Determination of the nature of nodules often relies on CT-enhanced scans, which, however, increase the radiation dose and contrast events, while plain scans alone fail to provide a qualitative diagnosis [22, 23].

Dual-source CT achieves the separation of iodine from the surrounding soft tissues and acquires information about the lesion [24]. Previous research has revealed a *U*-shaped association between iodine consumption and thyroid problems, as well as abnormal modifications in iodine metabolism in thyroid lesions [15–27]. DS-DECT detects the iodine content of thyroid nodules, and the iodine content in benign nodules exceeds that of malignant nodules, indicating that thyroid lesions have implications for follicular cells and the decreased iodine metabolism in the lesion area. Moreover, DS-DECT allows for in-depth analysis of the lesion by establishing iodine images [28]. Iodine uptake by thyroid follicular cells within thyroid nodules and adenomas is reduced in the presence of hyperplasia or degeneration of thyroid tissue or incomplete degeneration within the nodule; in malignant nodules, cellular heterogeneity within the lesion is more pronounced, and thyroid follicular cells have a reduced or even absent capacity for iodine uptake [29, 30]. The iodine content in follicular adenoma lesions is negative in malignant nodules and positive in benign nodules [31]. Therefore, the use of DS-DECT to analyze the iodine content of thyroid nodules enhances the accuracy of determining the benignity and malignancy of nodules [32]. In DS-DECT, two X-ray bulbs emit X-rays using different tube voltages, and the relevant information is collected using a detector, followed by the acquisition of the images after mathematical operations. In comparison to color ultrasonography, DS-DECT achieves chemical processing of chemicals, which increases the sensitivity of the examination and enhances the diagnostic effect on thyroid nodules [33, 34]. In the material separation of DS-DECT, the decay of iodine at different energies is available for an accurate diagnosis of thyroid nodules [35].

RETRACTED

In the present study, there was a significant difference in the iodine content of the lesioned solid tissue versus normal tissue, and a significant difference in the iodine content of malignant and benign nodules, suggesting that DS-DECT enhances the diagnostic accuracy of the malignancy of thyroid nodules and facilitates early treatment. The reason for this may be that the iodogram technique is an imaging technique that extracts iodine from the image based on the different attenuation trends of iodine at different energies under dual-energy CT scans compared to other tissues [36]. Dual-source CT dual-energy imaging iodogram measures the iodine content of thyroid nodules more accurately than a CT plain scan alone [37]. Moreover, in the venous phase, the NIC and standardized CT values of benign nodules were higher than those of malignant nodules, which was consistent with the results by Varghese [38]. Their findings showed lower iodine concentrations of malignant nodules than in benign nodules in the venous phase. This indicates that thyroid follicular cells in benign nodules uptake iodine, whereas in malignant nodules thyroid follicular cells are mostly substituted by cancer cells and connective tissue, which severely compromises iodine uptake capacity. In addition, the detection rate of malignant nodules with irregular morphology and calcification was higher than that of benign nodules, suggesting that benign nodules have clear borders with an intact envelope and no invasion into the surrounding normal thyroid tissue. The sensitivity and specificity of NIC differential diagnosis were 90.48% (38/42) and 88.89% (16/18), respectively, and the sensitivity and specificity of standardized CT value differential diagnosis were 92.86% (39/42) and 94.44% (17/18), respectively, as shown by the ROC curve. By the Kappa test, the differential diagnosis of NIC and standardized CT values in the venous phase was in high agreement with the morphological differential diagnosis (Kappa = 0.901, 0.883). This suggests that the iodine content of the thyroid lesion is available to determine the nature of the thyroid lesion preoperatively and to avoid overtreatment. The reason may be that dual-source CT is a quantitative identification of the iodine content of the iodogram by the different attenuation coefficients of two different energies on the substance, using iodine as the reference substance, which is the physical basis for the separation of dual-energy substances in dual-source CT [39, 40]. Therefore, by observing the iodine content of thyroid lesions, a quantitative indicator can thus be obtained, which allows for preoperative determination of the nature of the thyroid lesion to avoid overtreatment.

RETRACTED

## 5. Conclusion

DS-DECT is indeed highly accurate in determining the benignity and malignancy of thyroid nodules and yields a strong potential for clinical promotion to allow for prompt treatment.

## Figures and Tables

**Figure 1:** (a)–(d) is plain scan image, arterial phase image, venous phase image, and coronal MPR reconstruction of the thyroid gland image, respectively. Patient information: A 43-year-old female was admitted to the hospital with a left-sided thyroid mass found on physical examination for over 1 month. The thyroid ultrasound suggested a nodule in the left lobe of the thyroid gland with TI-RADS class 4a. CT showed a small nodular hypointense shadow in the left lobe of the thyroid gland with a maximum size of about 4.3 × 3.9 mm, which was progressively and significantly enhanced and was slightly hypointense compared with the surrounding normally enhanced thyroid gland, with indistinct demarcation. Postoperative pathology confirmed that the nodule was a papillary thyroid carcinoma.

**Figure 2:** (a)–(f) show the thyroid plain scan image, venous phase image, coronal MPR reconstruction image, iodine coverage image, dual energy image, and coronal iodine coverage image. Patient information: A 52-year-old female was admitted to the hospital with bilateral thyroid masses found on physical examination for 2 years. A multifocal cystic mass was found in the thyroid gland, with a large left lobe and TI-RADS grade 3. CT showed an enlarged left lobe of the thyroid gland with a round cystic low-density shadow of approximately 23 × 18 mm in size, with a clear border and uniform density, and a visible separation. No significant enhancement was seen in the cystic portion. The iodine image clearly showed the distribution of iodine in the compartment and allowed for quantitative measurement of iodine content, which resulted in the diagnosis of nodular goiter. The postoperative pathology confirmed that the “left thyroid mass” was a nodular goiter with hemorrhage and cystic changes.

RETRACTED

**Figure 3:** ROC curve of NIC and standardized CT for diagnosis of malignant thyroid nodules in the venous phase.

**Table 1:** Iodine content (mg/ml).

Group	*n*	Diseased solid tissues		Normal tissues	
		Range	Mean	Range	Mean
Benign nodules	42	−0.9–2.3	0.5 ± 0.2	1.4–4.4	2.1 ± 0.6
Malignant nodules	18	−2.4–0.9	0.1 ± 0.1	1.5–4.4	2.3 ± 0.4
*t-value*			3.750		0.607
*P value*			0.003		0.555

**Table 2:** NIC and standardized CT values for benign and malignant nodules.

Group	*n*	Arterial phase		Venous phase	
		NIC	Standardized CT values (HU)	NIC	Standardized CT values (HU)
Benign nodules	42	0.35 ± 0.05	0.33 ± 0.05	0.83 ± 0.12	0.87 ± 0.15
Malignant nodules	18	0.36 ± 0.07	0.32 ± 0.06	0.61 ± 0.08	0.64 ± 0.11
*t-value*		−0.627	0.668	7.112	5.854
*P value*		0.533	0.507	<0.001	<0.001

**Table 3:** Examination results.

Groups	*n*	Morphological irregularities	Lesions with clear boundaries	Calcifications
Benign nodules	42	8 (19.05)	42 (100.00)	30 (71.43)
Malignant nodules	18	10 (55.56)	0 (0.00)	5 (27.78)
*X* ^2^		7.997	60.0	9.878
*P value*		0.005	<0.001	0.002

## Data Availability

All data generated or analysed during this study are included in this published article.
